This article has been retracted.

# Variations in Stable Carbon Isotope Composition and Leaf Traits of *Picea schrenkiana* var. *tianschanica* along an Altitude Gradient in Tianshan Mountains, Northwest China

**DOI:** 10.1155/2014/243159

**Published:** 2014-11-04

**Authors:** Huiwen Zhang, Jianying Ma, Wei Sun, Fahu Chen

**Affiliations:** ^1^Key Laboratory of Ecohydrology of Inland River Basin, Cold and Arid Regions Environmental and Engineering Research Institute, Chinese Academy of Sciences, Lanzhou 730000, China; ^2^Key Laboratory of Western China's Environmental Systems (Ministry of Education), Lanzhou University, Lanzhou 730000, China; ^3^Dunhuang Gobi and Desert Ecological and Environmental Research Station, Cold and Arid Regions Environmental and Engineering Research Institute, Chinese Academy of Sciences, Lanzhou 730000, China; ^4^Department of Renewable Resources, University of Wyoming, Laramie, WY 82071, USA

## Abstract

To understand the morphological and physiological responses of leaves to changes in altitudinal gradients, we examined ten morphological and physiological characteristics in one-year-old needles of *Picea schrenkiana* var. *tianschanica* at ten points along an altitudinal gradient from 1420 to 2300 m a.s.l. on the northern slopes of the Tianshan Mountains in northwest China. Our results indicated that LA, SD, LPC, and LKC increased linearly with increasing elevation, whereas leaf *δ* ^13^C, LNC, Chla + b, LDMC, LMA, and N_area_ varied nonlinearly with changes in altitude. With elevation below 2100 m, LNC, N_area_, and Chla + b increased, while LDMC and LMA decreased with increasing altitude. When altitude was above 2100 m, these properties showed the opposite patterns. Leaf *δ* ^13^C was positively correlated with N_area_ and LNC and negatively correlated with SD and LA, suggesting that leaf *δ* ^13^C was indirectly controlled by physiological and morphological adjustments along altitudinal gradients. Based on the observed maximum values in LNC, N_area_, Chla + b, and LA and the minimum values in LMA and LDMC at the elevation of 2100 m, suggesting higher photosynthetic capacity and greater potential for fast growth under superior optimum zone, we concluded that the best growing elevation for *P. schrenkiana* var. *tianschanica* in the Tianshan Mountains was approximately 2100 m.

## 1. Introduction

Stable carbon isotope composition (*δ* ^13^C) provides an integrated measurement of internal plant physiological and external environmental properties influencing photosynthetic gas exchange over the time when the carbon was fixed [1, 2]. So applications using stable carbon isotopes have developed from initially categorizing photosynthetic pathways (C_3_, C_4_, and CAM) to evaluating more critical impacts of environmental conditions on leaf photosynthesis [3–9]. However, this application requires better understanding of relationships between carbon isotope composition and plant physiological and morphological characteristics.

As a result of variation in environmental factors, such as temperature, precipitation, photosynthetically active radiation, and atmospheric CO_2_ concentration along altitudinal gradients, changes in morphological and physiological traits and leaf carbon isotope composition in alpine plants are expected. Therefore, altitudinal gradients provide unique experimental opportunities to study morphological and physiological responses of plants to environmental factors, as well as relationships between leaf carbon isotope composition and leaf morphological and physiological characteristics [9–14].

In general, leaf *δ* ^13^C values of most alpine plants increased with increasing altitude [6, 7, 15–21]. However, a decrease in leaf *δ* ^13^C with increasing altitude [4, 5, 22] or no linear relationships between leaf *δ* ^13^C and altitude [17, 23–30] have also been reported. Variation in leaf *δ* ^13^C has been found in correlation with leaf morphological traits (leaf thickness, leaf area, stomatal density, etc.) [13, 14, 23, 28, 31] and physiological traits (stomatal conductance, carboxylation efficiency, leaf mass per unit area, leaf nitrogen concentration, etc.) [9, 11–13, 15, 24, 28, 32, 33] along the altitudinal gradients. These findings show that there is considerable variation in the response of leaf morphological and physiological relationships to environmental variability and thus impact on leaf *δ* ^13^C.

*Picea schrenkiana* var.* tianschanica*, one of the major species of alpine and subalpine forests in western China, forms pure forests in the northern slopes of the Tianshan Mountains. These forests play a very important role in preventing soil erosion and soil water loss, regulating climate, as well as maintaining ecological stability [34]. Previous studies suggested that the continuous distribution of* P. schrenkiana* var.* tianschanica* on the north slopes of Tianshan Mountains is a result of combined water-heat conditions [35–38]. However, this hypothesis has been lacking in support from morphological and physiological aspects. We studied leaf morphological and physiological characteristics, including leaf *δ* ^13^C, in* P. schrenkiana* var.* tianschanica* growing along an altitudinal gradient on the northern slopes of the Tianshan Mountain. Our objectives were (1) to survey leaf *δ* ^13^C values and leaf morphological and physiological characteristics in response to changes in altitude, (2) to analyze relationships between leaf *δ* ^13^C values and leaf morphological and physiological characteristics and test the hypothesis that leaf *δ* ^13^C values were determined indirectly by physiological and morphological adjustments with changing environmental factors along with altitude gradient, and (3) to identify a relative optimum zone for the growth of* P. schrenkiana* var.* tianschanica* along the altitudinal gradients.

## 2. Materials and Methods

### 2.1. Study Sites

In September 2007, ten sampling sites were selected at about 100 m elevation intervals along an altitudinal gradient from 1420 m to 2300 m (at elevation of 1420, 1505, 1622, 1757, 1850, 1962, 2045, 2110, 2240, and 2300 m) in the northern slopes of the Tianshan Mountains. Sampling sites were located between 83°04′41′′E and 87°12′54′′E longitude and 43°10′57′′N and 44°05′06′′N latitude. The slope of the sampling sites ranged from 10% to 40%. Altitude, latitude, and longitude of each sampling site were determined by GPS (Magellan GPS315, Magellan, USA). Meteorological data representing the areas from low to high altitude located within the Tianshan Mountains are provided in Table 1 [39, 40]. The soil was classified as mountain grey-brown forest soil.

### 2.2. Sampling and Ecophysiological Measurements

To minimize the age effects, we selected all the sampling trees with same approximate height of about 5 m tall. Five mature trees at each site were selected for leaf sample collection. One-year-old needles were collected randomly from the south side of the crowns. The needles were placed in plastic bottle and kept in liquid nitrogen. Needles from five selected trees (100 needles per tree) at each sampling site were divided into five groups for leaf physiological and morphological measurements. Following the rehydration procedure, the needles were cut from the stem and gently blotted with tissue paper to remove any surface water before measuring water-saturated fresh mass. The projected surface area (LA) was determined by an LI-3000A portable area meter (Li-Cor, Lincoln, NE). Stomatal densities (SD) were determined using a 200x magnification with a KEYENCE VHX-Z100R scanning electronic microscope (Keyence, Japan) as described by Hultine and Marshall [13]. To avoid variations of SD at the base or tip, SD near the middle of the needle was reported. Dry mass was determined after the needles were oven-dried for 48 h at 80°C. Dry mass and LA were then used to calculate leaf mass per unit area (LMA). Dry matter content (LDMC) was calculated as a percentage of dry biomass to the saturated needle biomass. Leaf nitrogen concentration per unit mass (LNC) of dried tissue was determined by a micro-Kjeldahl digestion system (KDH, Shanghai QianJian instrument Co., Ltd, China). Leaf phosphorus concentration per unit mass (LPC) was determined by vanadium-molybdenum yellow colorimetric analysis methods with a spectrophotometer (VIS-7220, Beijing Modern Rayleigh Instrument Co., Ltd, China). Leaf potassium concentration per unit mass (LKC) was determined by flame photometer (410, Sherwood, UK) [41]. Pigment contents (Chla + b) of other fresh needles were analyzed with an* N*,* N*-dimethylformamide (DMF) extraction spectrophotometer method [42]. Leaf nitrogen concentration per unit area (N_area_) was calculated by multiplying LNC by LMA.

### 2.3. Stable Carbon Isotope Composition Analysis

Stable carbon isotope composition (*δ* ^13^C) of dry needles was determined by an elemental analyzer (Flash EA 1112, Thermo Electron, USA) coupled to a Finnigan Delta + XP continuous flow inlet isotope ratio mass spectrometer (Thermo Finnigan, Bremen, Germany) in the Stable Isotope Laboratory, Key laboratory of Western China's Environmental Systems (Ministry of Education), Lanzhou University. The *δ* ^13^C values were expressed in per mil deviation relative to the Pee Dee Belemnite (PDB) standard [43]. Precision of repeated measurements of laboratory standards was <0.2‰.

### 2.4. Statistical Analysis

Normality of distribution and homogeneity of variance were checked before any further statistical analysis. The normality was checked by Shapiro-Wilk (sample size was less than 50). Homogeneity was done by test of homogeneity of variances. Differences in leaf *δ* ^13^C and other leaf traits among different positions along the altitudinal gradient were determined using one-way ANOVA (Table 2). Linear and nonlinear regression models were used to analyze the relationships between elevation and leaf traits (Figure 1). Pearson's correlation was applied so as to check the existence of relationship between two variables in this research (Table 3). And the relationships between altitude and soil properties also were investigated (Figure 2). All the analyses were carried out by SPSS Version 16.0 (SPSS Inc., Chicago, IL, USA).

## 3. Results

### 3.1. Characteristics of Leaf  *δ* ^13^C and Other Leaf Traits

Leaf *δ* ^13^C values ranged from −30.55‰ to −24.69‰, with a mean of −28.42‰. There were significant differences in leaf *δ* ^13^C (*P* < 0.001). And significant differences in LA, SD, LNC, LPC, LKC, Chla + b, LDMC, LMA, and N_area_ among* P. schrenkiana* var.* tianschanica* populations at different altitudes were also detected (*P* < 0.001) (Table 2).

### 3.2. Altitudinal Changes of Leaf  *δ* ^13^C and Other Leaf Traits

Leaf *δ* ^13^C varied nonlinearly with increasing altitude. LA, SD, LPC, and LKC increased linearly with increasing elevation, whereas LNC, Chla + b, LDMC, LMA, and N_area_ varied nonlinearly with changes in altitude (Figure 1). There was an approximate critical altitude for variations of morphological and physiological factors near 2100 m altitude. Below 2100 m, LNC, Chla + b, and N_area_ increased significantly with increasing altitude (Figures 1(d), 1(g), and 1(j)), whereas LDMC and LMA decreased significantly along the altitudinal gradients (Figures 1(h) and 1(i)). In contrast, when altitude was above 2100 m, these properties showed the opposite patterns. The maximum values of LNC (15.42 ± 0.38 mg*·*g^−1^), N_area_ (4.14 ± 0.28 g*·*m^−2^), and Chla + b (2.44 ± 0.37 mg*·*g^−1^) and the minimum values of LDMC (451.80 ± 6.28 mg*·*g^−1^) and LMA (252.33 ± 3.60 g*·*m^−2^) were obtained at an altitude of about 2100 m. Indeed, maximum LA, LPC, and LKC were also detected at 2100 m (Figures 1(b), 1(e), and 1(f)).

### 3.3. Relationships between Leaf  *δ* ^13^C and Leaf Traits

According to Table 3, it showed that correlations between two variables were determined using Pearson's correlation. Leaf *δ* ^13^C was positively correlated with LNC and N_area_, while the correlation with LNC was medium (*r* = 0.550) and the correlation with N_area_ was weak (*r* = 0.422 and *r* = 0.397, resp.). Leaf *δ* ^13^C was negatively correlated with LA and SD, while the correlations were weak (*r* = −0.436 and *r* = −0.432, resp.). There was no significant relationship between *δ* ^13^C and LPC, LKC, Chla + b, LDMC, and LMA. In addition, it showed the weak (±0.31~±0.50) or medium (±0.51~±0.70) or strong (±0.71~±0.90) correlation between other leaf traits.

## 4. Discussion

### 4.1. Changes in Leaf Morphological and Physiological Traits along the Altitudinal Gradient

Leaf physiological and morphological traits of most alpine plants are strongly affected by different abiotic factors along altitudinal gradients. Low-altitude plants have to withstand the unfavourable climatic conditions of dry habitats, high temperatures, harsh radiation, and scant precipitation. On the other hand, high altitude plants have to face the adverse conditions with low temperatures accompanied by high irradiance, unavailable soil water, strong wind, and high vapor pressure deficits. So alpine plants show great phenotypic plasticity and adjust their morphology and physiology in response to surrounding environment.

In our study, with water-heat conditions turned better, SD increased linearly with increasing elevation (Figure 1(c)). Increases in SD with increasing altitude may compensate for the reduction in CO_2_ partial pressure [44] or may be associated with an improved efficiency in carbon dioxide uptake [45]. Increasing drought from lower to higher altitudes is considered to be the main stress force for changes of SD because of the fact that colder soil could reduce water uptake of root system and induce water stress [46]. LA, LPC, and LKC increased significantly with increasing altitude (Figures 1(a), 1(e), and 1(f)). But when altitude was above 2100 m, they all dropped slightly. At low altitude, heat stress, cold stress, drought stress, and high-radiation stress all tend to lead to relatively small leaves [47]. Moreover, low temperatures at high altitude might limit cell expansion. Phosphorus availability in the soil was higher, and leaf potassium content followed a similar pattern to soil total potassium content (Figure 2); this suggested that a large proportion of phosphorus and potassium in leaves might be taken up from the soil. When conditions become severe at higher elevation,* P. schrenkiana* var.* tianschanica* might allocate more phosphorus and potassium to protective tissues by osmoregulation to adapt to the native habits.

Our results showed that LNC, Chla + b, LDMC, LMA, and N_area_ varied nonlinearly with changes in altitude. There was an approximate critical altitude for variations of leaf traits near 2100 m altitude. Below 2100 m, LNC, Chla + b, and N_area_ increased with increasing altitude (Figures 1(d), 1(g), and 1(j)), whereas LDMC and LMA decreased along the altitudinal gradient (Figures 1(h) and 1(i)). In contrast, when altitude was above 2100 m, these properties showed the opposite patterns. Photosynthetic capacity generally increases with leaf nitrogen content because photosynthetic enzymes such as rubisco contain large quantities of N [13]. Moreover, photosynthetic pigments changing with increasing altitude can also reflect variation in photosynthesis ability [48]. We observed similar patterns in the variation of chlorophyll contents, LNC, and N_area_ along the altitudinal gradients. Similar results were reported in other conifer trees [25, 28]. Increasing chlorophyll contents, LNC, and N_area_ before 2100 m might be an adoption to increasing light intensities because assimilation rates in* P. schrenkiana* var.* tianschanica* were highly determined by light intensities [49]. In addition, nitrogen content increased with the altitude; the most likely explanation was that the large amount of nitrogen in leaves was taken up from the soil. This was consistent with our investigation of soil nitrogen supply (Figure 2). We found that LMA was higher at lower and higher altitudes but decreased at midaltitudes just as LDMC. The higher LMA probably results from higher temperatures and summer drought at lower altitudes [50] and cold temperature at higher altitudes [44, 51]. The effect of air temperature was even greater than the effect of water availability [46]. On the other hand, it has been pointed out that leaves with high LMA have a structure that reduces not only photosynthetic rates but also water losses by transpiration [13]. Leaves with high LDMC tend to be relatively tough and are thus assumed to be more resistant to physical hazards which are often observed in plants growing in highly disturbed environments [47].

### 4.2. Impacts of Variation in Leaf Morphological and Physiological Traits on Leaf  *δ* ^13^C

The present study found that LNC and N_area_ showed positive correlation with leaf *δ* ^13^C (Table 3). Levels of N in plant tissues have been reported to have a positive correlation with altitude, and this increase in leaf nitrogen content with altitude may increase CO_2_ demand at the sites of carboxylation and progressively result in higher carboxylation efficiency [12, 33, 48, 52]. A primary explanation for altitudinal trends in leaf nitrogen content is that low temperatures and short growing seasons at high elevation reduce growth rate and might consequently have a concentrating effect on leaf nitrogen content [48, 52]. High leaf nitrogen concentrations make increased investment in leaf chlorophyll and rubisco possible [53], and this in turn may cause high carboxylation efficiencies and high leaf *δ* ^13^C value [11, 12, 33]. We therefore concluded that leaf nitrogen content was one of influencing factors on variation in leaf *δ* ^13^C values along the altitudinal gradients.

Generally, LA decreases linearly with altitude [11, 47, 54, 55]. However, some studies also have found that LA increases with altitude [56] or initially increases and then decreases again [25, 28]. Plants often have larger LA at midelevation where temperature and precipitation may be optimal [28] and the large size of leaves with high nitrogen concentration can fix more CO_2_ potentially than smaller leaves [12]. And this might lead to high carboxylation efficiencies or high photosynthetic capacities which induced high leaf *δ* ^13^C value. In our study, LA negatively correlated with leaf *δ* ^13^C (Table 3). Similar results have been reported by Zhao et al. [28]. The findings show there is remarkable variation in the response of LA to environmental hydrothermal conditions, and thus impact on leaf *δ* ^13^C.

Stomata allow water loss by transpiration and the entry of CO_2_ into the leaf for photosynthetic carbon fixation. We observed that SD in* P. schrenkiana* var.* tianschanica* increased linearly with altitude (Figure 1; *r* = 0.752), and there was a negative relationship between *δ* ^13^C and SD (Table 3). Similar results were observed in conifer trees [25, 28]. Earlier publications demonstrate that an increase in atmospheric CO_2_ results in a decrease in SD of plants [5]. Körner and Cochrane [57] considered that SD generally increases with altitude and presumably increases the diffusive supply through the stomata. Stomatal conductance increases the supply of CO_2_ to the interior of the leaf and would be expected to reduce *δ* ^13^C of fixed carbon. So increases in SD should reduce, rather than enhance, *δ* ^13^C composition of leaves with altitude. This discrepancy leads to the suggestion that the SD was not the key to understanding carbon isotope trends with altitude [13]. It might be that the stomata growing at higher altitude could not open entirely under severe environmental conditions. Our study suggested that the variation in SD was not the major cause of the observed increase in *δ* ^13^C with altitude. Some other morphological and physiological factors along with the altitude should have an integrated influence on *δ* ^13^C values.

### 4.3. Optimum Growing Zone

For a single species that exhibits a continuous distribution over a broad elevational transect, there must be a relative optimum zone for growth [58]. The physiological potential for vigorous growth and relatively high photosynthetic rate might decrease below or above that optimum altitude. Leaf area, leaf nitrogen content, chlorophyll contents, LMA, LDMC, and so forth often change remarkably at this altitude [24, 25, 28].

Leaf area has important consequences for the leaf energy and water balance and relates to climatic variation, geology, altitude, and latitude. Along with altitude gradient, leaf size variation can also be linked to both temperature and water availability. On average, heat stress, cold stress, drought stress, and high-radiation stress all tend to lead to relatively small leaves [47]. The small size of leaves from high elevations might result in a lost opportunity for carbon fixation [12]. At their optimal midelevation, plants often have larger LA [25, 28], potentially fixing more CO_2_ [12].

LDMC can be used to predict species position along a resource-use gradient [47, 59] and is related to the average density of the leaf tissues and tends to scale with LMA. Furthermore, LDMC has been shown negatively with potential relative growth rate or mass-based maximum photosynthetic rate [47]. Leaves with high LDMC tend to be relatively tough and are thus assumed to be more resistant to physical hazards (e.g., wind and hail), while leaves with low LDMC tend to be associated with high productivity, which is often observed in plants growing in highly disturbed environments [47].

LMA can be thought of as the investment (leaf mass) associated with a given potential rate of return (light-capture area) [60]. Low LMA, indicating greater potential for fast growth (higher rate of return on a given investment) and enhanced nutrient investment [60], tends to have higher photosynthetic capacity per unit leaf mass, resulting from having larger light-capture area deployed per mass, higher leaf N concentration [61, 62], and shorter diffusion paths from stomata to chloroplasts [63]. Species in resource-rich environments tend to have low LMA [47], while high LMA has been shown to be advantageous in low-resource environments or harsh situations [64].

In the Tianshan Mountains, rainfall varies nonlinearly with elevation. Maximum annual precipitation is obtained at midelevation. Temperature decreases with increasing elevation [38]. Early studies indicated that there existed relatively more suitable environmental conditions for growth of* P. schrenkiana* var.* tianschanica* in the middle of their distribution region [35]. In their superior environment, plants had a relatively high photosynthetic rate and growth rate. In our study, LNC, N_area_, chlorophyll contents, and LA increased significantly with increasing altitude, and they reached the maximum values at an altitude of about 2100 m. At the same time, LMA and LDMC decreased in better conditions with respect to elevation, and they reached the minimum values at an altitude of about 2100 m. All these changes suggested higher photosynthetic capacity and greater potential for fast growth under lower utilization of resources [60, 62]. However, climatic conditions become severe and soil becomes barren at lower and higher elevation. And these bad environmental conditions will cause a direct restriction of leaf expansion, accompanied by reduced leaf nitrogen content and chlorophyll contents, and LMA and LDMC increased indicating potential advantages in low-resource environments or an increase in resistance to harsh situations [60, 64].

## 5. Conclusions

The results of our research suggested that there are evident altitudinal variation and substantial plastic responses in morphological and physiological characteristics of* P. schrenkiana* var.* tianschanica* across environmental gradients. Reversible physiological and morphological responses allowed plants to adapt to changing water-heat conditions and soil conditions with increasing elevation. In addition, *δ* ^13^C was positively correlated with N_area_ and LNC and negatively correlated with SD and LA. This reinforced the hypothesis that leaf *δ* ^13^C of* P. schrenkiana* var.* tianschanica* was indirectly controlled by physiological and morphological adjustments along altitudinal gradient. Moreover, based on the observed maximum values in LNC, N_area_, Chla + b, and LA and the minimum values in LMA and LDMC at the elevation of 2100 m, suggesting higher photosynthetic capacity and better growth, the 2100 m elevation zone appeared to be an optimum habitat for* P. schrenkiana* var.* tianschanica*.

## Figures and Tables

**Figure 1:** Variation in (a) leaf stable carbon isotope composition (*δ* ^13^C), (b) leaf projected area per 100 needles (LA), (c) stomatal density (SD), (d) leaf nitrogen concentration per unit mass (LNC), (e) leaf phosphorus concentration per unit mass (LPC), (f) leaf potassium concentration per unit mass (LKC), (g) pigment contents (Chla + b), (h) leaf dry matter content (LDMC), (i) leaf mass per unit area (LMA), and (j) leaf nitrogen concentration per unit area (N_area_) in* P. schrenkiana* var.* tianschanica* along the altitudinal gradients.

**Figure 2:** Relationships between altitude and soil properties (values are means ± standard deviation).

**Table 1:** Meteorological data of located stations within the research area.

Station	Latitude	Longitude	Time (yr.)	Altitude (m)	Mean annual temperature (°C)	Mean annual precipitation (mm)
Urumchi	43°78′	87°65′	1961–2000	935	6.8	265
Xiaoqüzi	43°29′	87°06′	1971–2000	1872	2.3	542
Tianshan forest ecosystem research station	43°26′	87°28′	2005-2006	1905	2.0	573
Houxia	43°29′	87°07′	1978–2002	2350	1.5	445

**Table 2:** Significance of the altitudinal effects on leaf traits.

	*δ* ^13^C (‰)	LA (cm^2^)	SD (number*·*mm^−2^)	LNC (mg*·*g^−1^)	LPC (mg*·*g^−1^)	LKC (mg*·*g^−1^)	Chla + b (mg*·*g^−1^)	LDMC (mg*·*g^−1^)	LMA (g*·*m^−2^)	N_area_ (g*·*m^−2^)
SS	25.4	696.4	42.6	260.7	262.0	246.1	39.4	30341.9	9292.0	17.4
MS	2.8	77.4	4.7	29.0	29.1	27.3	4.4	3371.3	1032.4	1.9
*F*	27.7	196.6	40.8	66.9	190.9	185.9	22.4	27.2	24.2	53.7
*P*	<0.001	<0.001	<0.001	<0.001	<0.001	<0.001	<0.001	<0.001	<0.001	<0.001

**Table 3:** Correlation coefficients among leaf traits.

	*δ* ^13^C (‰)	LA (cm^2^)	SD (number*·*mm^−2^)	LNC (mg*·*g^−1^)	LPC (mg*·*g^−1^)	LKC (mg*·*g^−1^)	Chla + b (mg*·*g^−1^)	LDMC (mg*·*g^−1^)	LMA (g*·*m^−2^)	N_area_ (g*·*m^−2^)
*δ* ^13^C (‰)	1									
LA (cm^2^)	−0.436^*^	1								
SD (number*·*mm^−2^)	−0.432^*^	0.590^**^	1							
LNC (mg*·*g^−1^)	0.550^**^	0.313^*^	−0.146	1						
LPC (mg*·*g^−1^)	−0.049	0.813^**^	0.428^**^	0.542^**^	1					
LKC (mg*·*g^−1^)	0.222	0.681^**^	0.514^**^	0.618^**^	0.848^**^	1				
Chla + b (mg*·*g^−1^)	0.135	0.596^**^	0.032	0.694^**^	0.738^**^	0.648^**^	1			
LDMC (mg*·*g^−1^)	0.305	−0.582^**^	−0.094	−0.260	−0.594^**^	−0.403^**^	−0.618^**^	1		
LMA (g*·*m^−2^)	−0.231	−0.576^**^	−0.177	−0.601^**^	−0.741^**^	−0.706^**^	−0.521^**^	0.313^*^	1	
N_area_ (g*·*m^−2^)	0.397^*^	0.463^**^	0.002	0.962^**^	0.602^**^	0.675^**^	0.735^**^	−0.340^*^	−0.618^**^	1

^*^ *P* < 0.05; ^**^ *P* < 0.01.
